# A Novel Piano Arrangement Timbre Intelligent Recognition System Using Multilabel Classification Technology and KNN Algorithm

**DOI:** 10.1155/2022/2205936

**Published:** 2022-07-09

**Authors:** Yuan Lu, Chiawei Chu

**Affiliations:** ^1^Academy of Music, Yuxi Normal University, Yuxi 653100, China; ^2^Faculty of Data Science, City University of Macau, Macau 999078, China

## Abstract

In this paper, melody and harmony are regarded as the task of machine learning, and a piano arranger timbre recognition system based on AI (Artificial Intelligence) is constructed by training a series of samples. The short-time Fourier transform spectrum analysis method is used to extract the piano timbre characteristic matrix, and the electronic synthesis of timbre recognition is improved by extracting the envelope function. Using the traditional multilabel classification method and KNN (K-nearest neighbor) algorithm, a combined algorithm of these two algorithms is proposed. The experimental results show that the detection rate increases from 61.3% to 70.2% after using the combined classification algorithm. The correct rate also increased from 40.3% to 48.9%, and the detection rate increased to 74.6% when the K value was set to 6. The experimental results show that, compared with the traditional classification algorithm, this algorithm has a certain improvement in recognition rate. Using this system to recognize the timbre of piano arrangement has a high recognition accuracy, which is worthy of further popularization and application.

## 1. Introduction

The art of music is vast and profound; for a true pianist or piano educator, touching the tip of the iceberg of piano music works is insufficient; they must also broaden their horizons to include all aspects of music art. It is obvious that you can hear the sounds of various instruments when playing the digital recording of the piano concerto. People may not be able to correctly identify the names of some instruments, but they should be able to recognize their general categories, such as stringed or wind instruments. The loss of information such as bells, melodies, and ringtones will have a significant impact on the accuracy of music recovery results, resulting in low recovery efficiency. The development of contemporary electronic music has been aided by the rise of AI (Artificial Intelligence) technology [1], and the technology's application fields are constantly expanding. The use of AI technology to solve problems like timbre recognition and feature extraction in music arrangers has gotten a lot of attention.

The exploration and research in the field of music have developed rapidly with the progress of computer science. Nowadays, the digital music creation mode has completely changed the traditional music industry and greatly improved the quality and production efficiency of music works. Patil and Elhilali recognized music as a series of music fragments, analyzed their music styles, and then established a statistical model in the existing music database to predict the style classification of other music [2]. Aucouturier and Pachet defined the emotional attribute value as an emotional plane and proposed a fusion algorithm, considering that a piece of music may have multiple emotions with interval changes [3]. Kailash et al. introduced the recognition principle of machine auditory system and applied the heuristic processing method to the sound signal, which can preliminarily understand the sound signal [4]. Chen and Guo put forward a timbre model based on piano pronunciation waveform, which uses the spectrum characteristics and amplitude envelope characteristics of timbre to construct piano timbre model [5]. Wu et al. introduced a timbre model based on trapezoidal wave. The model is divided into two parts: vibration submodel and inclusion submodel. Time, asymmetry, trapezoidal degree, and three angles are defined as timbre parameters for timbre synthesis [6]. A series of research works have been made on multipart piano music, and a machine hearing system has been developed, which can recognize multipart piano music. In the research process of machine hearing, the frequency spectrum analysis of musical instrument timbre signal has always been a research hotspot, which requires the selection of frequency spectrum feature extraction technology. Different technical application fields and analysis results are different.

The AI-based piano arranger timbre recognition system separates harmonic signals at the edge of music, transmits timbre, analyzes timbre signal continuity, and implements the system design, but the system's performance is poor. It is demonstrated that timbre is a type of sound feature that includes frequency spectrum and time based on psychological judgments of music timbre, analysis of physical characteristics of sound, and research of machine learning methods. To fully comprehend the true meaning of timbre, it is necessary to fully comprehend the number and significance of characteristic parameters that affect timbre. As a result, to design a piano arrangement timbre recognition system based on AI, this paper uses the Fourier analysis method. The use of computer technology in the field of music, as well as the use of computer technology in the field of music, will provide mankind with new musical experiences.

The innovation of this paper is summarized as follows:

1. In this paper, taking piano music signal recognition and synthesis as an example, the characteristics of piano music signals are recognized and analyzed by mathematical methods, and the extracted characteristics of piano music signals are digitized to realize piano timbre recognition and simulation.
2. Using the multilabel classification method [7, 8] and KNN algorithm, a combined algorithm of these two algorithms, namely, ML_KNN classification algorithm, is proposed. The experimental results show that the recognition rate of the classification algorithm based on ML_KNN is higher than that based on multilabel decision tree.

The following is a list of the sections of this article: The first section discusses the research's background and significance before moving on to the paper's main work. The second section focuses on the related timbre recognition techniques used in piano arrangements. The third section outlines the research's specific methods and methods of implementation. The superiority and feasibility of this research model are confirmed in the fourth section. The summary of the full text is found in the fifth section.

## 2. Related Work

### 2.1. Timbre Feature Recognition Method

Musical instrument timbre recognition is an important research trend of machine hearing. However, from the academic point of view of machine hearing, the difficulty of musical instrument timbre recognition is roughly equal to that of speech recognition. However, scholars who study musical instrument recognition need to be proficient in both music and computer, so the research population is small, and the progress of musical instrument timbre recognition is slower than that of speech recognition, with few achievements and few references.

Mitrovic et al. adopted KNN (K-nearest neighbor) method and Gaussian mixture model to realize automatic classification of musical instrument features. The experimental results show that the highest recognition rate of 14 musical instruments is 90% [9]. Peretz et al. extracted a series of musical sound features that can be perceived by human auditory system from the musical sounds of 27 musical instruments and applied these features to the classification of musical instruments. Finally, the recognition rate of musical instrument perception difference reached 71%, and the system developed by them had good stability in dealing with reverberation and noise syllables [10]. The music composition system developed by Han et al. allows people without music skills to intervene in its composition system to create music, and the generated melody can reach 16 bars in length [11].

Xing et al. pointed out that when using genetic algorithm to solve melody harmony, we will encounter the problem of harmony search space in irrelevant local optimal area [12]. Omar et al. put forward a graph [13] of arranging very interesting harmony for a given melody based on the training data. This graph model may be better than the hidden Markov model in obtaining the root sound movement showing global correlation. Wang et al. think that the timbre space of musical instruments includes five dimensions, and besides the characteristic dimensions of time domain and frequency domain, it also includes the dimension of time-frequency combination [14].

### 2.2. Research Status of Multilabel Classification

A natural scene can contain multiple target objects. For example, the scene can be described with multiple class labels. They usually use multiple labels to train samples to solve problems. However, this method is not suitable for music database, because each instrument can play different notes, and some of them can express different timbres by using different playing skills.

Xiang et al. discussed the emotion classification in music clips, which involved six kinds of emotion classification labels and a small number of timbre feature values. Emotion is a higher level of information, which can be further obtained from pitch, volume, rhythm, and timbre [15]. Mancia and Janssen used the trained neural network to recognize and classify 166 groups of music samples and achieved good classification results [16]. Cerri et al. proposed a pitch-independent instrument recognition system [17]. Further extracting features including basic frequency, spectrum, time domain, and modulation and solving their respective multivariate normal distributions, the recognition rate of the final instrument family reaches 90%, and the recognition rate of a single instrument reaches 80%. Sering et al. proposed several methods for high-order statistical modeling of musical sound signals and evaluated them in the environment of multimedia sound retrieval [18]. Ju et al. made it possible to separate two or more musical instruments by using single channel speech separation method through Gaussian modeling [19].

The multilabel emotion classification method based on dictionary is to extract the emotion keywords from the text on the basis of emotion dictionary database, so as to classify the text. Yong et al. designed a chat system based on text and embedded conversation messenger emotion estimation. This system is based on an emotional content evaluation module that evaluates text chat messages, extracts related emotions from the text through keywords, and then evaluates the text emotions through syntactic features, speech synthesis, and related emotional gestures [20]. Yan et al. put forward an interdisciplinary approach to study the structure of emotion and society, analyzed the influence of society on cognition and emotional interaction, examined how emotions are stimulated and expressed in society, and studied how society affects the processing and regulation of emotions [21].

## 3. Methodology

### 3.1. Piano Arrangement Timbre Recognition

#### 3.1.1. Piano Spectrum Analysis

Timbre is the basis of identifying musical instruments, and it is the characteristic information that distinguishes musical instruments from other musical instruments. The sound of an instrument consists of fundamental tone and overtone. It is the tone with the lowest pitch frequency, and those that are not pitch are collectively called overtones. The human auditory system can tell which musical instrument the sound comes from, because the high-frequency harmonic components of musical instruments are different, and the harmonic proportions of different musical instruments are also different. The definition of timbre is too subjective to lead to automatic classification of music. Therefore, the main work of this paper is to parameterize the timbre features in detail for automatic recognition and classification.

Piano arrangers must play the parts of multiple people at the same time, which necessitates exceptional performance skills. The piano arranger represents the combination of conductor and orchestra, and the orchestra is made up of multipart staff. It is necessary to use both hands to play the condensed version of the previous parts. The band's concert editing is moderately difficult and plays a major and minor role in the overall work; the reduction of band accompaniment is relatively simple. Because the accompaniment part usually does not have a lot of “scenes,” it is usually only used to fill in the gaps in the solo and highlight the band's characteristics.

Even if the strength, position, and striking method are all the same for piano strings, the volume is not always the same. Through simple music training, humans can tell the difference between musical instrument timbres. Humans can quickly distinguish piano tones from the sounds of a variety of musical instruments as well as background noise. To achieve musical instrument timbre recognition by listening machine, we must first understand the mathematical principle of sound waves and then determine the differences between musical instrument timbres in mathematical expression and then use these differences to quickly identify and distinguish musical instrument timbres. The projection function is used to represent the low-dimensional features of the spectrum after the rank reduction:

(1) $$\begin{array}{c} y_{t}=\left[r_{t},{\tilde{x}}_{t}^{T}v_{1},{\tilde{x}}_{t}^{T}v_{2},\text{…},{\tilde{x}}_{t}^{T}v_{k}\right], \end{array}$$

where $r_{t},{\tilde{x}}_{t}^{T},v_{1},\text{…},v_{k}$ is calculated by the spectrum basis function.

The resonance frequency of different instrument resonators is different, and the shape of resonance peak in frequency spectrum is also different. Not only is resonance peak the decisive factor of sound quality, but also it reflects the physical characteristics of the resonant cavity. Cepstrum coefficient is a method to express resonance peak.

The cepstrum coefficient containing the signal quantity *y*(*n*) is defined as *F*, and *F* represents discrete Fourier transform.

(2) $$\begin{array}{c} c\left(n\right)=F^{-1}\left\{\text{log}|F\left\{y\left(n\right)\right\}\right\}. \end{array}$$

The analysis of MFCC (Mel frequency cepstrum coefficient) is based on human auditory mechanism; that is, the spectrum of speech is analyzed according to the results of human auditory experiments, in the hope of obtaining good speech characteristics [17]. The delineation of the frequency domain of human subjective perception is not linear, and there is the following formula:

(3) $$\begin{array}{c} F_{mel}=1125\;\log\;{\left(1+\frac{f}{700}\right)}_{V}, \end{array}$$

where *F*_*mel*_ is the perceived frequency in Mel; *f* is the actual frequency in Hz.

The process of extracting MFCC features includes the following steps:

1. Input the audio signal to be processed.
2. Select the window length *N* to preemphasize, frame, and window the input audio signal.
3. The processed audio segments of each frame are subjected to FFT (fast Fourier transform) to obtain the corresponding frequency spectrum.
4. Mel cepstrum is obtained according to formula (3).
5. Take the logarithm of Mel frequency cepstrum and do inverse Fourier transform (get Mel frequency cepstrum coefficient MFCC), and the 2nd–13th coefficients after discrete cosine transform are MFCC coefficients.

The lowest frequency of the piano is 28.5 Hz, so it can be seen that all the sound bands of the piano remain in the Fourier transform analysis area. Based on the auditory nervous system, human ears can fully perceive the music spectrum and feel the timbre of piano, so the choice of spectrum structure analysis is actually a simulation of human auditory nervous system. Based on Matlab software, according to the principle of Fourier transform, the FFT function program is written, and the spectrum analysis diagram of single tone is obtained. It shows that there are multiple octave overtones and octave vibrations in the piano, and the uniqueness of the piano and the rich characteristics of piano timbre are expounded.

#### 3.1.2. Extraction of Timbre Matrix

Strings are the piano's basic sound source. The player presses the keys to cause the hammer to strike the strings, causing the strings to vibrate and producing the original sound, which then causes the resonance system to resonate. Some researchers discovered that some functional waveforms resemble those found on the piano. Sinc, Gaussian, and Cauchy functions are examples of specific functions that can be selected. The frequency domain waveform of piano tones can also be approximated using these specific functions, according to the researchers. Choose a suitable piano accompaniment type metastructure from the existing library, and configure the piano accompaniment spectrum for the new melody using the modes of melody segments, the root of chords, and various permutation functions provided in the selected piano accompaniment type metastructure.

In order to improve the high-frequency resolution of music signal and analyze the whole spectrum of the whole frequency band, a processing method is proposed, which usually uses a first-order digital filter for preemphasis before signal extraction. The transfer function of this filter is expressed as

(4) $$\begin{array}{c} H\left(z\right)=1-\alpha z^{-1}. \end{array}$$

In the above formula, *α* is the preemphasis factor, which is generally taken as a decimal close to 1. In this paper, it is taken as 0.95. Preemphasis process transforms the signal as follows:

(5) $$\begin{array}{c} x\left(n\right)=x\left(n+1\right)-\alpha x\left(n\right). \end{array}$$

The data obtained from the above formula is the preemphasized data, where *x*(*n*) is the original audio signal.

In the calculation of short-time autocorrelation function detection method, multiple multiplications lead to a large amount of calculation, while the average amplitude difference method with long and short time uses a simpler difference form, which avoids multiple multiplications and achieves a performance similar to autocorrelation function.

The short-time average amplitude difference function *F*_*n*_(*k*) of the audio signal *s*(*m*) is defined as follows:

(6) $$\begin{array}{c} F_{n}\left(k\right)=\sum_{m=0}^{N-k-1}\left|S_{n}\left(m+k\right)-S_{n}\left(m\right)\right|. \end{array}$$

In the above formula, *N* represents the window length added by the audio signal *s*(*m*); *S*_*n*_(*m*) is defined as follows:

(7) $$\begin{array}{c} S_{n}\left(m\right)=s\left(m\right)w\left(n-m\right). \end{array}$$

The process of estimating pitch frequency by short-time average amplitude difference function detection method includes the five following steps:

1. Input the audio signal to be processed.
2. The input audio signal is preprocessed by windowing, framing, and endpoint detection, so that the audio signal of each frame becomes a short-term stable signal.
3. Calculate the short-term average amplitude difference function of each frame signal, and get the valley value of the pitch period position.
4. The obtained valley value estimates the pitch period and calculates the inverse of the pitch period to obtain the pitch frequency.

Because the weighted Cauchy function waveform is close to the piano waveform and can describe the fundamental frequency and frequency doubling analysis, and the simulation effect is similar to the actual timbre, the fifth frequency doubling method is selected to simulate and extract the piano timbre. Assume that the discrete Fourier transform of the discrete event signal *x*(*m*), namely, *X*(*iλ*), can be expressed as

(8) $$\begin{array}{c} X_{j}\left(i\lambda \right)=T_{j}\left(i\lambda \right)*P_{j}\left(i\lambda \right),\\ T_{j}\left(i\lambda \right)=\left\{\begin{array}{cc} B_{j}\frac{b_{j}}{b_{j}^{2}+{\left(\lambda -\lambda_{j}\right)}^{2}}, & \lambda_{j}-b_{j}\leq \lambda \leq \lambda_{j}+b_{j},\\ B_{j}\frac{2}{\left|\lambda -\lambda_{j}\right|}, & \text{Other}. \end{array}\right) \end{array}$$

In the above formula, *λ*_*j*_ represents the fundamental frequency or frequency multiplication of *j* sound; *B*_*j*_ represents amplitude; *b*_*j*_ stands for adjusting the waveform width around *λ*_*j*_; *P*_*j*_ stands for sine and cosine function, which accurately simulates playing timbre, intensity, and pitch to realize computer performance.

The basic idea of KNN (K-Nearest Neighbor) is as follows: according to the traditional vector space model, the text content is formalized as a weighted feature vector in the feature space. For a test text, calculate its similarity with each text in the training sample set, find out *K* most similar texts, and judge the category of the test text according to the weighted distance. According to the feature words, a test text vector is formed. Calculate the text similarity between the test text and each text in the training set, and the calculation formula is

(9) $$\begin{array}{c} \text{Sim}\left(d_{i},d{}_{j}\right)=\frac{\sum_{k=1}^{M}W_{ik}\times W_{jk}}{\sqrt{\sum_{k=1}^{M}W_{ik}^{2}}\sqrt{\sum_{k=1}^{M}W_{jk}^{2}}}, \end{array}$$

where *d*_*i*_ is the feature vector of the test text and *dj* is the center vector of class *j*; *M* is the dimension of the feature vector; *W*_*k*_ is the *k*-th dimension of the vector.

In the *k* neighbors of the test text, calculate the weight of each class in turn, and the calculation formula is as follows:

(10) $$\begin{array}{c} P\left(X,C_{j}\right)=\left\{\begin{array}{cc} 1, & \sum_{d_{i}\in KNN}\text{Sim}\left(x,d_{i}\right)y\left(d_{i},C_{j}\right)-b\geq 0,\\ 0, & \text{Other,} \end{array}\right) \end{array}$$

where *x* is the feature vector of the test text; *Sim*(*x*, *d*_*i*_) is the similarity calculation formula; *b* is the threshold, which needs to be optimized; and the value of *y*(*d*_*i*_, *C*_*j*_) is 1 or 0. If *d*_*i*_ belongs to *C*_*j*_, the function value is 1; otherwise, it is 0.

In this chapter, KNN algorithm is improved. By introducing multilabel classification, an extended KNN algorithm, namely, ML_KNN (multilabel k-nearest neighbor) classification algorithm, is proposed to further improve the efficiency of classification matching. ML_KNN algorithm is the realization of this paper based on ML_KNN classification. The algorithm is as follows:

1. Divide the audio file of chord music into divided frames with index window of 1 s.
2. 12 MPEG eigenvalues and 72 new time domain eigenvalues are extracted.
3. *N* tags with the highest confidence are selected as candidate tags for the current frame, and other tags with low confidence are discarded.
4. After all the individual frames in the index window are classified, the average confidence of each candidate instrument tag is calculated, and if the average confidence is greater than the optimal threshold parameter, the candidate tag is retained. Otherwise, it will be discarded.

To sum up, the flow chart of piano arrangement timbre recognition is shown in Figure 1.

Using self-developed amplitude feature extraction code, the relationship between amplitude and time of sine wave, piano, flute, and guitar music is analyzed, and the envelope function of different instruments is determined to be different. With a good envelope function, we can simulate the sound intensity and amplitude characteristics of wind instruments and stringed instruments and even the subtle differences between percussion instruments and plucked instruments.

### 3.2. System Implementation

The sound library generation module, which includes the piano arrangement sound recognition system, is the system's core module. This module generates the piano sound library in the audio system using the audio synthesis model and recognizes the timbre of the piano arrangement using the audio data provided by the sound acquisition module and the timbre parameters provided by the man-machine interaction module. Different timbre parameters can be used to generate different piano timbres. A computer-based sound library generation module is used to realize the piano arrangement timbre recognition system in the application experiment for this document's sound library generation. The system is modular in design and has a high degree of versatility, with modules such as audio file reading and writing, audio information analysis, timbre parameter acquisition, and timbre and simulation performance. The general architecture of piano arrangement pitch recognition system is shown in Figure 2.

In piano simulation function module, piano can play different types of music and opera scores, which is widely used and can act as a band, so piano is the best choice for playing musical instruments. Piano timbre editing function module can record timbre editing in various ways in detail; in particular, the music timbre editing with wide range is difficult, but timbre editing is very critical. The acquisition module edits and acquires the timbre parameters through the man-machine interface. The timbre synthesis module is used for synthesizing timbre files, supporting batch synthesis of various timbres, and displaying the synthesis progress in real time. The simulation performance module is used to assess the simulation performance of timbre or music.

The unique piano timbre obtained from the recording is determined by the vibration equation of the strings, and the amplitude energy changes from strong to weak, so it cannot be processed twice. On the other hand, the monophonic amplitude of electronic synthetic piano is stable, and the loudness does not change. In the postprocessing, envelope function can be added to control the change of amplitude, so as to reproduce the difference between hitting strength and delaying pedal and make music more emotional. Here, the pitch variable in the metastructure of the piano accompaniment sound mode can be determined. If some notes in the metastructure are imitated, their pitch is related to the pitch of the original melody being imitated.

## 4. Experiment and Results

We can build a data prediction model by machine learning algorithm and automatically identify the emotional features of music by computer. From the dataset of 400 pieces of music, we selected the feature data of 300 pieces of music as the training set (80% of the data as the training set and 20% as the test set) and the feature data of the other 100 pieces of music as the test set. When using ML_KNN, the training set is cross-validated, so as to obtain the optimal values of the parameters in the model. Finally, we tested the model, and the specific results of model comparison are shown in Figures 3 and 4.

The average correlation coefficient (CC) for the test set is 45.36 percent. The test set's MSE (mean squared error) is 0.038. It can be seen that the ML_KNN algorithm performs better in terms of musical emotional cognition. However, recognition rates for three emotions, Modest, Dream, and Graceful, are all very low in the test set, indicating that more research is needed. Correlation is a general method that is independent of the stream because it is done in the audio domain. This eliminates the tedious task of parsing the text's outline. This function can clearly reflect the intensity change of sound at different times during the arrangement process. It is possible to ensure that the pitch synthesis process of a piano arrangement is essentially consistent with the changing trend of tone using the envelope function extraction. This function is performed while removing some unwanted noise. This method can be used in practice indefinitely. If the processing is done in a professional lab with a well-configured computer cluster, it can achieve extremely high efficiency while saving time and money.

The frequency composition and proportion of synthetic timbre and real timbre are different (the proportion of harmonic amplitude coefficient is also different), so the two timbres are different in theory, which is proved by listening timbre. Compared with the positions surrounded by squares in Figure 4, although the synthesized timbre is very smooth in time domain, there are many burrs in frequency domain, and the timbre shows great noise. Therefore, their frequency domain characteristics are quite different. The single-tone datasets of musical instruments are classified, and the timbre expression spectrum is compared and analyzed based on the harmony structure proposed in this paper, so as to find the characteristics that can best reflect the timbre of musical instruments. Split the mono dataset of the instrument into five different datasets. The classification results based on different timbre features in different musical instrument monophonic datasets are shown in Table 1 and Figure 5. In the experiment, KNN is used as the classifier, the training set is 4/5 of the experimental data, and the test set is 1/5 of the experimental data.

It can be seen that the recognition rate of dataset 1 is generally high, because the timbre features of dataset 1 are all within a certain range, and the recognition of a single instrument is to find the specific corresponding point within this range. Regardless of the type of function set on which MFCC is based, the timbre expression spectrum of this paper performs well. According to the timbre expression spectrum function, the recognition rate of dataset 1 reaches 91.5%. According to MFCC function, the recognition rate of dataset 2 is 95.2%, that of dataset 3 is 78.4%, that of dataset 4 is 94.1%, and that of dataset 5 is 92.6%, which is the best result.

Extracting the same combination features of timbre and based on four supervised pattern recognition algorithms, KNN, Naive Bayes, Decision Tree, and ML_KNN, the classification and recognition experiments of single tones of musical instruments are carried out, respectively. The results are shown in Table 2 and Figure 6.

As can be seen, ML_KNN has the highest recognition rate across all datasets, so ML_KNN is chosen as the classifier for musical instrument classification and recognition in this paper. In addition, KNN is second only to ML_KNN in terms of classification and recognition of musical instruments. The performance of a detuned mode oscillator is better than that of a critical mode oscillator in various networks, which can be attributed to the clamping phenomenon mentioned earlier. The process of hijacking between local oscillator groups in the network to better track the time can be thought of as the rhythm change of a piece of music. The oscillator will show similar frequencies in the local area where strong resonance occurs. Average field networks have higher evaluation indices than other networks, but they also have a higher standard deviation. This demonstrates that the results of each round in the cross-validation process vary widely.

We conclude from our timbre analysis that all frequency components in the frequency domain interact to form a rich piano timbre and that synthesis of piano timbre cannot rely solely on overtone frequency components. The ratio of the vibration frequencies of the two pitches that make up the intervals determines the harmony of intervals, which is a characteristic that reflects the basic properties of intervals. Concordant intervals sound good and blend together, whereas dissonant intervals sound rougher and do not blend together. The Fourier transform algorithm is used to calculate the frequency, amplitude, and phase of various sine wave signals by accumulation [18]. Different playing skills of many musical instruments can produce different timbres. MFCC is extracted from these single-frame musical instrument sounds by describing the standard equation. The frame size is 130 ms, and the overlapping size of two adjacent frames is 80 ms, which reduces the information loss caused by window function. The hop count of the frame is 45 ms. The classifier is trained on these feature databases.  Figure 7 shows the comparison results of ring estimation based on multilabel classifier.

It can be concluded that, after introducing ML_KNN classification algorithm, the label Decision Tree classification algorithm with more prediction effects is obviously improved. After using ML_KNN classification algorithm, the detection rate is increased from 61.3% to 70.2%. The correct rate also increased from 40.3% to 48.9%. When the *k* value was set to 6, the detection rate increased to 74.6%, but the correct rate decreased to 41.2%. The conclusion of this experiment is that ML_KNN classification algorithm has better recognition effect than Decision Tree classification algorithm.

In the process of learning and studying music scores, pianists will naturally find a lot of music knowledge to supplement, such as musical instrument materials, pronunciation principles, staff of various transposed musical instruments, orchestration methods, and performance methods. To shorten the spectrum of vocal music, we need to know the pronunciation methods. No matter what note it is, the same attenuation rate is used, but, through the judgment of human ears, it can be found that the noise is reduced but not eliminated, so the music played is not very effective, and it is not musical with fluctuations. The combination of piano timbre characteristic matrix and sound intensity envelope curve can effectively distinguish the timbre differences of different songs, that is, identify the timbre of piano arrangement.

## 5. Conclusions

To sum up, this paper designs an AI-based piano arranger timbre recognition system based on Fourier analysis. Through short-time Fourier frequency shift spectrum analysis, the ringing characteristic matrix can be extracted. Get a tone shift envelope curve. The piano timbre can be clearly identified by the timbre characteristic matrix and transposition envelope curve. ML_KNN classification algorithm is applied to timbre recognition of chord music. The experimental results show that ML_KNN classification algorithm can improve the accuracy of chord music timbre recognition. After using ML_KNN classification algorithm, the detection rate increased from 61.3% to 70.2%. The correct rate also increased from 40.3% to 48.9%, and the detection rate increased to 74.6% when the *k* value was set to 6. The experimental results show that the timbre recognition system designed in this paper can synthesize clear piano music and has good timbre recognition performance, which is worthy of wide application.

## Figures and Tables

**Figure 1:** Flow chart of piano arrangement timbre recognition.

**Figure 2:** Overall architecture of piano arrangement timbre recognition system.

**Figure 3:** MSE test results of music emotion cognitive model.

**Figure 4:** CC test results of music emotion cognitive model.

**Figure 5:** Single-tone classification results of musical instruments.

**Figure 6:** Classification and recognition results of musical instrument tones.

**Figure 7:** Comparison results of timbre estimation of multilabel classifiers.

**Table 1:** Single-tone classification results of musical instruments based on different timbre features.

Dataset number	Frequency domain characteristics	Time domain characteristics	MFCC	Timbre expression spectrum
1	43.2	62.1	87.4	91.5
2	25.6	37.4	95.2	90.2
3	22.1	52.1	78.4	75.6
4	40.6	49.3	94.1	88.5
5	23.9	47.7	92.6	91.6

**Table 2:** Classification and recognition results of musical instrument tones based on different classifiers.

Dataset number	KNN	Naive Bayes	Decision Tree	ML_KNN
1	94.3	62.5	86.9	97.2
2	95.1	74.9	88.2	98.3
3	83.2	51.2	56.2	88.9
4	93.6	75.1	90.1	96.8
5	94.5	60.6	91.3	97.4

## Data Availability

The data used to support the findings of this study are available from the corresponding author upon request.
